The article "Analysis of Cervical Spine Alignment Change after Modified Kurokawa Cervical Laminoplasty in the Patients with Cervical Myelopathy and Straight Cervical Spine" was published in 2021. Journal: Biomed Res Int.

# Analysis of Cervical Spine Alignment Change after Modified Kurokawa Cervical Laminoplasty in the Patients with Cervical Myelopathy and Straight Cervical Spine

**DOI:** 10.1155/2021/6658766

**Published:** 2021-01-21

**Authors:** Shangbin Cui, Fuxin Wei, Xizhe Liu, Shaoyu Liu

**Affiliations:** ^1^Guangdong Provincial Key Laboratory of Orthopedics and Traumatology, The First Affiliated Hospital of Sun Yat-sen University, Guangdong, China; ^2^The Seventh Affiliated Hospital of Sun Yat-sen University, Guangdong Province, China

## Abstract

Laminoplasty is widely used to decompress the spinal cord in patients with multilevel cervical lesions. Straight cervical alignment may not be a good candidate for laminoplasty because of postoperation progression of kyphosis and loss of cervical spine range of motion (ROM). However, clinical outcomes of laminoplasty did not show a strong and consistent effect based on cervical sagittal alignment. Moreover, the kyphosis progression and ROM change after operation for the patients with preoperative strange cervical alignment are still unclear. This study is to evaluate the change of cervical alignment and ROM in patients with straight cervical alignment after modified Kurokawa cervical laminoplasty. Thirty patients with multiple-level cervical spondylosis (CSM) and straight cervical alignment were included. All patients underwent laminoplasty with the reconstruction of the spinous process-ligament-muscular complex (SPLMC). The modified JOA score was analyzed for clinical assessment. The change of cervical alignment, ROM, T1 slope, and intervertebral disc space Cobb angle were analyzed for radiological assessment. The average JOA score at preoperative and 2 years follow-up were 7.8 ± 1.4 and 13.6 ± 2.1, respectively. The recovery ratio was 63%. At the 2 years follow-up, there were 18 patients who acquired lordotic cervical alignment. 10 patients remained as straight cervical curve, and 2 patients' cervical alignment developed mild kyphosis. 28 out of 30 patients showed improvement of cervical alignment. The cervical alignment was improved from 1.29 ± 10.04° preoperative to 9.58 ± 8.65° postoperative. However, the ROM decreased from 36.8 ± 18.92 preoperative to 25.08 ± 12.10° postoperative. A positive correlation was found between the C2/4 angle change and cervical alignment change, T1 slope and cervical alignment, cervical alignment, and neutral position flexion reserved ROM. A negative correlation was found between the C1/2 angle change and cervical alignment change. Laminoplasty with a reconstruction of SPLMC followed by appropriate postoperative muscle exercises may be an encouraging way to maintain or improve physiological alignment and prevent postoperation kyphosis deformity for the CSM patients with straight cervical alignment at 2 years follow-up.

The article "Analysis of Cervical Spine Alignment Change after Modified Kurokawa Cervical Laminoplasty in the Patients with Cervical Myelopathy and Straight Cervical Spine" was published in 2021. Journal: Biomed Res Int.

## 1. Introduction

Degenerative diseases of the cervical spine are increasing among the geriatric population, and surgical treatment is becoming more common [1]. Double door laminoplasty has been widely used to treat patients with myelopathy due to cervical intervertebral disc herniation, spinal canal stenosis, and multiple-segment ossification of the posterior longitudinal ligament ossification. This surgical technique preserves the integrity of the posterior bone-ligament structure, meanwhile maintains the stability immediately after surgery [2]. However, this procedure invades the cervical posterior muscular-ligament complex, and it can inevitably disturb the cervical sagittal balance [3].

The ideal result after surgery is to recover the blood flow of the decompressed spinal cord through nerve decompression via effective posterior migration of the spinal cord. Previous studies showed that cervical sagittal alignment plays an important role in the clinical outcomes of laminoplasty. If the patient's lordotic alignment of the cervical spine is well maintained, the outcome of the surgery is always good [4]. On the other hand, the straight or kyphotic curvature of the cervical spine is not recommended as a good indication for laminoplasty because the laminoplasty may not create enough posterior migration of the spinal cord. Long-term results of conventional laminoplasty have shown a significant incidence of postoperative kyphotic deformity and loss of ROM [4, 5]. However, recent studies showed that preoperative cervical sagittal alignment did not have a consistent effect on the clinical outcomes of laminoplasty. The patients with straight or mild cervical kyphosis may also be suitable for laminoplasty [6–8]. Kim et al. [9] reported that radiological and clinical outcomes were compared after laminoplasty between the group of patients who had cervical kyphosis with Cobb angle < 10° and the cervical lordosis group. He found that there was no significant difference between the two groups.

In this regard, the authors hypothesize that by properly maintaining and reconstructing the spinous process-ligament-muscle complex (SPLMC) during laminoplasty surgery, followed by postoperative muscle strengthening exercises, the formation of kyphosis can be decreased and even the preoperative mild kyphotic or straight alignment can be improved. Moreover, the spinal cord may have enough posterior migration for the ideal clinical outcomes. By analyzing the changes of cervical spine radiological parameters, this study intends to confirm whether the straight alignment of the cervical spine would also be a proper indication for laminoplasty.

The article "Analysis of Cervical Spine Alignment Change after Modified Kurokawa Cervical Laminoplasty in the Patients with Cervical Myelopathy and Straight Cervical Spine" was published in 2021. Journal: Biomed Res Int.

## 2. Materials and Methods

### 2.1. General Data

From January 2018 to October 2020, 30 consecutive patients (18 males, 12 females) with a mean age of59.2 ± 17.6 (range 43 to 75 years old) were recruited. Patients diagnosed with cervical spondylosis myelopathy (CSM) with unhealthy cervical alignment (straight) were recruited into this study. All the patients underwent modified Kurokawa laminoplasty with SPLMC reconstruction back in situ before October 2018. Patients were asked to wear a Philadelphia cervical orthosis collar for 3 weeks. The patients who had cervical segmental instability, local kyphosis, prominent anterior compression, spinal injury, infection, revision surgery, tumor, and inflammatory arthritis were excluded. All surgeries were performed by the same senior experienced surgeon. The follow-up period was at least 2 years (range from 2.3 to 2.5 years).

### 2.2. Radiologic Evaluation

In all patients, pre- and postoperative, 2 years follow-up AP view plain radiographs of the cervical spine were obtained, as well as dynamic flexion-extension lateral radiography. Different time points plain radiographs were analyzed in comparison to identify changes in the curvature of the cervical spine, changes in the range of motion (ROM) of the neck, cervical spine alignment, and T1 slope angle.

The cervical alignment was determined by measuring the angle formed by two lines extending from the inferior borders of the second and seventh cervical bodies in the neutral position. On dynamic films, the ROM of the cervical spine was evaluated by the summation of the cervical Cobb angle in flexion and in extension. The angle of intervertebral disc space (IVDA) was expressed as the angle between two lines extending from the inferior margin of the upper vertebra and the superior margin of the lower vertebra. The positive value of cervical lordosis meant lordosis, and the negative value meant kyphosis. Cervical alignment configurations were classified into four groups: lordotic, straight, kyphotic, and sigmoid as described by Toyama et al. [10] (Figure 1). In our study, we only selected the patients with a straight curve.

The following parameters were investigated including the pre- and postoperative C2-C7 Cobb angle, change in cervical alignment, the constitution of cervical alignment in each intervertebral disc space, C2-C7 range of motion (ROM), the constitution of ROM in each intervertebral disc space, the cervical flexion reserved ROM in the neutral position, T1 slope change, C2-C7 SVA, and the correlation between different parameters. The parameters were calculated with the following formula:

Cervical alignment changes (°) = (postoperative C2 − C7 Cobb angle) − (preoperative C2 − C7 Cobb angle), 

IVD space ROM (°) = (extension IVD space Cobb angle) − (flexion IVD space Cobb angle), 

C2 − C7 ROM (°) = (extension C2 − C7 Cobb angle) − (flexion C2 − C7 Cobb angle), 

Neutral position flexion reserved ROM (NFRROM) (°) = (neutral C2 − C7 Cobb angle) − (flexion C2 − C7 Cobb angle).

The article "Analysis of Cervical Spine Alignment Change after Modified Kurokawa Cervical Laminoplasty in the Patients with Cervical Myelopathy and Straight Cervical Spine" was published in 2021. Journal: Biomed Res Int.

Two independent observers measured each parameter on images; the measurements were obtained using electronic calipers by using the Surgimap software (Nemaris, Inc.). In the present study, we investigated the reliability of the measurement techniques and found good to excellent intra- and interobserver agreement for each parameter (Kappa > 0.70).

### 2.3. Operative Technique

All laminoplasties were performed by the double-door (midsagittal spinous-splitting) technique [11]. Under general anesthesia, Mayfield three points head fixator is fixed to the cranium of a patient and connected to the operation table with the cervical spine slightly flexed. Care must be taken not to hyperextend the cervical spine at the time of setting. After identifying the level of C2 and C7 spinous processes by touching them over the surface of the skin, a central longitudinal skin incision is made. The nuchal ligament is centrally incised not to damage the posterior branch of the cervical nerve. By detaching the paravertebral muscles from each spinous process and maintaining the interspinous ligaments, the laminae from the caudal side of C2 to the cranial side of C7 (or C6) are exposed. We use the modified Kurokawa double-door laminoplasty technique. C3 spinous process and lamina was removed, and the ligamentum flavum are also resected to decompress the spinal cord. Laminae were exposed to the medial border of the facet joints, where bilateral longitudinal grooves were made with a high-speed burr. Both the side inner lamina cortices were preserved. The spinous process was meticulously split with a thin fretsaw. A laminoplasty spreader was used to open the spinous process symmetrically. When the upper end of laminoplasty was C3, the semispinalis cervicis was taken caution in order not to be detached from the C2. The split spinous processes were opened bilaterally. At each level, the shape of the widened space is trapezoidal both on the axial and frontal sections. A trial spacer is placed into the widened space, and an appropriate size of the real spacer is selected. A 2 mm hole to accommodate a thread for fixing the spacer is made at about 8 mm or more superficial from the inner plate of the lamina. Spacers made of hydroxyapatite were held in position by tying them to split spinous process by nonabsorbable sutures. After the laminoplasty is done, the Mayfield three-point head fixator is adjusted to the cervical alignment with a lordotic curve. All of the detached insertion of the posterior paraspinal muscles was sutured back with the original spinous process after the elevation [12]. Then, we sutured the supraspinal ligament and interspinal ligament with bilateral paraspinal muscles (such as trapezius, splenius capitis, semispinalis capitis, semispinalis cervicis, and multifidus). By using the nonabsorbable sutures, we make a reconstruction connection between the reconstructed spinous process and adjacent process-ligament-muscle complex. Finally, suture the nuchae ligament back in situ by continuous stitching and form a complete tension band for the posterior extension muscle which was needed for the lordotic cervical alignment. The schematic diagram is shown in Figure 2.

The article "Analysis of Cervical Spine Alignment Change after Modified Kurokawa Cervical Laminoplasty in the Patients with Cervical Myelopathy and Straight Cervical Spine" was published in 2021. Journal: Biomed Res Int.

All patients were allowed to ambulate on the second postoperative day using a walker or wheelchair with wearing a soft neck collar. At the end of 1 month postoperatively, the collar is removed. For the first 6 months, isometric neck muscle exercises were performed. Patients were advised to perform three to six sets of 10–50 extension repetitions (held for approximately 30 seconds to 1 minute in the maximal extension position) every day. Patients were educated to gradually increase the intensity of their muscle exercises. In general, the patients were expected to exercise at roughly 75% of their maximal intensity. As expected, the intensity of this exercise regimen varied from patient to patient. A typical case is shown in Figure 3.

### 2.4. Clinical and Radiology Assessment at Follow-Up

Their neurological conditions were assessed using the Japanese Orthopedic Association (JOA) scoring system proposed by the Japanese Society of Spinal Surgery. Recovery ratio was calculated using Hirabayashi's formula: recovery ratio (%) = (postoperative JOA–preoperative JOA/17–preoperative JOA)^∗^100%, with a recovery rate of 100% indicating the best postoperative improvement. Postoperative radiographs were taken at the end of 2 years follow-up. X-rays and computed tomographic scans were also done as needed before these dates if the patient had any significant complaints. The JOA scores were also acquired before surgery and at follow-ups.

### 2.5. Statistical Analysis

Data are presented as mean ± standard deviation and calculated using the IBM SPSS Statistics 20. Each independent variable of subjects was compared between preoperation and 2 years after operation using the independent *t*-test for continuous variables. To assess correlations between independent variables and the dependent variable, we used Spearman correlation coefficients. Variables with a *P* value less than 0.10 in univariate analysis were considered for multivariate linear analysis. Adjusted odds ratios (ORs) with 95% confidence intervals (CIs) are presented with their respective *P* values. A value of *P* < 0.05 was accepted as significant.

The article "Analysis of Cervical Spine Alignment Change after Modified Kurokawa Cervical Laminoplasty in the Patients with Cervical Myelopathy and Straight Cervical Spine" was published in 2021. Journal: Biomed Res Int.

## 3. Results

### 3.1. Clinical Assessment

The average blood loss is 95 ± 24.5 ml. The average operation time is 80 ± 19.7 min. The mean preoperative JOA scores were 7.80 ± 1.4. At one-year follow-up, the average JOA scores were 13.6 ± 2.1. The JOA recovery rate is 63.0 ± 15.7%. There was a statistically significant difference between preoperative and postoperative JOA scores (*P* < 0.05). None of the patients had axial symptoms or C5 palsy at the last follow-up.

### 3.2. Changes of Radiology Parameters

On the computed tomographic scan, all patients had maintained the “open door” of laminoplasty and the hinge site of the lamina reached the bony fusion. On the X-ray, there were 30 patients defined as straight cervical preoperation. At the 2 years follow-up, there were 18 patients who acquired lordotic cervical alignment. 10 patients remained as straight cervical curve and 2 patients' cervical alignment developed mild kyphosis. The details of cervical radiological parameter changes are shown in Table 1.

### 3.3. Correlation Analysis between Different Parameters

Correlation analysis showed that there were different correlation relationship between C1/2 angle, C2/4 angle, ROM, C2/4 ROM, T1 slope, cervical alignment, and NFRROM. The correlation analysis is shown in Table 2.

### 3.4. Comparison of IVD Space Alignment and ROM according to Preoperative T1 Slope

Based on the previous studies by Lin et al., T1 slope may have an influence on the cervical alignment. Patients with low T1 slope or compensated condition are suitable candidates for laminoplasty [13]. We subdivided the patients into two categories according to the preoperative T1 slope > 20 degrees [13]. Group 1 (14 patients) showed T1 slope > 20 degrees. Group 2 (16 patients) showed T1 slope < 20 degrees. The IVD space alignment and ROM in the two groups are shown in Figure 4. Change in IVD space cervical alignment was significantly different between the two groups at the C2/3 level. Group 1 was higher than group 2. Change in IVD space ROM was significantly different between the two groups at C4/5 and C5/6 levels. Group 1 showed a negative change. However, Group 2 showed a positive change. The other IVD space ROM also showed a negative change.

The data was presented as mean ± SD, “^∗^” means *P* < 0.05, and there was a significant statistical difference between groups.

The article "Analysis of Cervical Spine Alignment Change after Modified Kurokawa Cervical Laminoplasty in the Patients with Cervical Myelopathy and Straight Cervical Spine" was published in 2021. Journal: Biomed Res Int.

## 4. Discussion

Double-door laminoplasty is an effective surgical method and widely used for the treatment of patients with cervical spondylosis, spinal canal stenosis, and multiple-segment ossification of the posterior longitudinal ligament (OPLL). The cervical motion can be maintained by preserving the posterior neck structure and achieves indirect posterior decompression.

Both preoperative and postoperative cervical lordosis are considered perquisites for successful outcomes. The adequate decompression can be obtained when cervical lordosis is maintained, allowing the posterior shift of the cervical spinal cord after laminoplasty. Clinical improvement after laminoplasty may be unsatisfactory if the focal kyphosis angle is larger than 13° [14] or if the thickness of ossification of posterior longitudinal ligament exceeds the line that connects the midpoints of the spinal canal at C2 and C7 (K-line) [15]. On the other hand, studies also showed that kyphosis within 10° of cervical kyphosis has no different postoperative outcome from the cervical lordosis after laminoplasty [9]. There is a dispute in treating the patients with a straight, mild kyphotic, or sigmoid cervical alignment, and the results of cervical alignment changes have been unclear and inconclusive. In our study, these kinds of patients received laminoplasty, and the JOA score was improved from 5.80 ± 1.4° preoperative to 13.6 ± 2.1° at 2 years follow-up which proved that the laminoplasty has good clinical efficacy.

The original concept of laminoplasty was to reconstruct the bony structure of the posterior cervical spine. Previous reports showed that laminoplasty prevented postoperative kyphotic deformity [16]. Unfortunately, patients who undergo laminoplasty tend to exhibit a postoperative change towards kyphotic alignment despite having sufficient lordosis preoperatively. Long-term results by Satomi et al. [17] showed that open-door laminoplasty decreased cervical alignment only 1.5° (transformed from Ishihara's index to the C2-C7 angle) in patients with cervical spondylotic myelopathy at a 5-year postoperative period. With regard to change in cervical alignment, the literature reported a wide range of values, from a 7° loss of lordosis after 29 months of follow-up to 16.7° gain of lordosis in a separate study after 9 months of follow-up [18, 19]. The mean preoperative and postoperative C2-7 angles (available for 2470 patients) remained stable from 14.17°(±0.19°) to 13.98° (±0.19°) of lordosis (average follow-up time 39 months) [19]. Reviews which focused on the mean preoperative and postoperative C2–7 angles or curvature index numbers showed that 28.8% of the studies reported stable alignment, 45.0% of the studies reported worse kyphosis (i.e., a mean decreased C2–7 angle or curvature index), and 26.3% reported increased kyphotic curve [19]. The maintaining of normal posterior elements of the cervical spine also plays an important role in the normal physiological curve. The results of the simulation analyses showed that the primary cause of postlaminectomy deformity was the resection of one or more spinous processes and such posterior ligaments as ligament flava and supraspinous and interspinous ligaments. After the removal, the tensile stresses that were distributed through the posterior ligaments before the surgery were transferred to the facets, leading to an imbalance of the stresses on the spinal bodies and causing the deformity [20]. Destruction of facet joints or joint capsule also can follow kyphosis and ligaments, and muscles are also regarded as tension bend against flexion force [21]. The surgery method had been improved to preserve or reconstruct them as much as possible. Studies found that postoperative kyphosis has been observed to develop in 6% to 46% of patients after conventional laminectomy [22, 23], but 0% to 10% of patients after laminoplasty with reattachment of the cervical extensor musculature [24, 25]. Other authors suggested posterior element–sparing or restriction of the laminoplasty from techniques [26, 27], C3 to C6 instead of C-7 to reduce kyphosis [28]. Reduced surgical exposure and no detachment of the semispinalis cervicis muscle from the C-2 spinous process or avoiding the C-2 lamina in total have also been claimed to be associated with favorable results in regard to postoperative kyphotic changes [29]. In our study, an effort was made to preserve muscle attachment as much as possible and reconstruct all the flexion muscle back after the laminoplasty trying to regain as many functional muscles as possible. The cervical alignment improved from 1.29 ± 10.04° preoperatively to 9.58 ± 8.65° 2 years follow-up. The changes in IVDA change also showed a significant difference from C2/3 to C5/6 (range from 3.08 ± 5.05° to 3.96 ± 7.90°).

The article "Analysis of Cervical Spine Alignment Change after Modified Kurokawa Cervical Laminoplasty in the Patients with Cervical Myelopathy and Straight Cervical Spine" was published in 2021. Journal: Biomed Res Int.

The reduction of cervical spine ROM after laminoplasty was also noted in previous studies. An overall mean (calculated from 2390 patients) of 47.3% loss of ROM was reported [30]. The mean follow-up period also influenced the loss of ROM in the studies; a smaller degree of loss of ROM was shorter (mean follow-up time 32 months) than that in the studies with a >25% loss of ROM (mean follow-up time 54 months) [30]. Some authors have reported a relationship between cervical ROM and cervical posterior muscle condition, especially that of deep muscles after laminoplasty [31]. In addition, modified surgical techniques have been developed to preserve the paraspinal muscles not only to maintain cervical ROM but also to reduce axial symptoms [12, 32]. In our study, we made a similar observation: The ROM was reduced from 36.8 ± 18.92° preoperatively to 25.08 ± 12.10° at 2 years follow-up by 31%. The significant difference was found in IVD space ROM change at C2/3, C3/4, C4/5, and C6/7 (range from −2.67 ± 6.03° to −4.15 ± 6.11°). This suggested that this change could be the result of the stripped muscles which attached to the spinous process and articular capsule. However, after a period of muscle exercise, the situation in most patients improved. It seems that shorter bed rest and cervical orthosis and early neck ROM exercises result in less restriction of ROM in the long term [33].

Results in many clinical studies indicate that alterations of spinal curvature are important factors determining a poor clinical outcome. The loss of lordotic curve and kyphotic deformity may result in the persistence of adverse stresses applied to the underlying neural structures. Moreover, such changes may restrict disengagement of the spinal cord from anterior compressive lesions, with the resulting persistence of adverse stresses acting on the cord [34]. The straight curve is a protective change against the spinal and cord from anterior compression in the cervical spondylosis. Consequently, if the nerve compression is progressed, the kyphotic cervical alignment can develop. One of the reasons for kyphotic change is that the spinal canal and the intervertebral foramina may increase in size when in kyphosis status. Holmes et al. demonstrated that the change in the volume of the spinal canal between C2 and C7 showed a linear relationship with the angle of flexion and the dynamic canal width [35]. However, in the late stage, kyphotic changes could not offer enough relief for the continued compression on the spinal cord, and the nerve function will eventually be damaged. In our study, we found that the preoperative cervical alignment had a negative correlation with C1/2 angle change (*r* = −0.4499, *P* = 0.0465) and a positive correlation with preoperative T1 slope (*r* = 0.3972, *P* = 0.0297). This may reflect the cervical spine self-adjustment process when mild cervical alignment happens. And we also found that the postoperative cervical alignment was negatively correlated with the postoperative C1/2 angle (*r* = −0.4771, *P* = 0.0334), positively correlated with postoperative T1 slope (*r* = 0.4063, *P* = 0.0259), and postoperative NFRROM (*r* = 0.5171, *P* = 0.0034).

After the laminoplasty and reconstruction of posterior SPMLC, the harmonious state was achieved. The cervical alignment is no longer compensated by the C1/2 angle but also by the other IVD space. Cervical alignment change also has a positive correlation with C2/4 angle change (*r* = 0.8086, *P* = 0.0046) and negative correlation with C2-C7 SVA (*r* = −0.3442, *P* = 0.0015). We inferred that during the laminoplasty, the C3 posterior elements were removed, and because of that, there is more space for C2-C4 moving segments. With the improvement of cervical alignment, the center of the C2 vertebral move backward and the C2-C7 SVA decrease.

The article "Analysis of Cervical Spine Alignment Change after Modified Kurokawa Cervical Laminoplasty in the Patients with Cervical Myelopathy and Straight Cervical Spine" was published in 2021. Journal: Biomed Res Int.

The cross-section of the cervical spine and layers of nuchal muscles were as follows: the trapezius in the 1st layer, the splenius in the 2nd layer, and the semispinalis capitis in the 3rd layer of the nuchal ligament. Semispinalis cervicis and multifidus are attached to the sides of the spinous process. In our surgery, we intend to remove the spinous process and lamina of C3 to provide more space for the C2 spinous process to move backward and prevent the reconstructed C3 spinous process impinged on the flexion muscle attached to the C2 spinous process. In the final step of recombination, Mayfield three-point head fixator was adjusted to maintain the cervical spine with a lordotic alignment. Then, the flexor muscles were sutured back to the original attachment. The continuous suture of the nucha ligament would make the ligament tighter and shorter than the original one. And in this way, the cervical alignment will maintain or improve. The SPMLC includes the spinous process, supraspinous and interspinous ligaments, and associated muscles. The SPLMC is an important part of the posterior column of the spine. It is required to maintain a normal physiological cervical curve [36]. One solution to avoid the development of postoperative kyphosis is to recover the tension by preserving the spinous process and the interspinalis muscles as a support like kotoji and resuturing the semispinalis cervicis muscles that had earlier been detached from the C2 spinous process before wound closure [11]. The repair of muscular attachment to the part of the spinous process helps to maintain the blood supply and preserve muscle volume which is important to maintain cervical lordosis. Studies showed that the method in which all the posterior muscle attachment is preserved (myoarchitectonic spinolaminoplasty) resulted in the least loss of lordosis [37]. Kato et al. [12] reported a series in which the detached insertion of the posterior paraspinal muscles was sutured back with the original spinous process after the elevation and the clinical outcomes were good.

The sagittal alignment plays an important role in the pathogenesis of CSM and assessment of the spinal structure; including global spine balance and cervical regional alignment is necessary to make a clinical decision. Kim et al. proposed 1 hypothesis—the same degree of cervical lordosis might have a different meaning according to the degree of T1 slope. They announced that patients with high T1 needed more cervical lordosis to maintain equilibrium. Therefore, cervical alignment could be within the compensated or uncompensated condition. It is important to assess each patient based on the individual condition of global sagittal balance and regional alignment. Laminoplasty itself results in damage of the posterior muscular-ligament complex and disrupts original cervical alignment. To compensate for this problem, the global spine will make corresponding adaptation to reestablish the postoperative equilibrium between whole spine sagittal balance and cervical regional alignment [13].

The article "Analysis of Cervical Spine Alignment Change after Modified Kurokawa Cervical Laminoplasty in the Patients with Cervical Myelopathy and Straight Cervical Spine" was published in 2021. Journal: Biomed Res Int.

In our study, the T1 slope changed from 22.25 ± 6.28° preoperatively to 20.71 ± 3.78° 2 years follow-up. T1 slope flexion angle remained the same, but the T1 slope extension angle changed from 21.20 ± 5.92° to 17.61 ± 7.51°. According to the T1 slope, we subdivided the patients into two groups. Group 1 with T1 slope > 20° had higher IVD space alignment change at the C2/3 level (*P* < 0.05) and minus the change in IVD space ROM change at C4/5 and C5/6 levels. However, Group 2 with T1 slope < 20 had a positive change in IVD space ROM change at C4/5 and C5/6 levels. We also found that in the postoperative IVD space cervical alignment, Group 1 showed lordotic alignment at C2/3, C4/5, C5/6, and C6/7. The group remained negative at C2/3, C4/5, and C6/7.

There are several limitations to this study. Firstly, the sample size is relatively small and lack of control group; the further study would be multicenter, large-scale trials to analyze the cervical alignment change after laminoplasty. Secondly, patients with cervical myelopathy can present with wide variation in the degree of involvement; further studies with matched controls may be necessary to predict the outcome of this type of surgery. Finally, the cervical deep extensor muscle plays an important role in maintaining cervical alignments; in this study, we mainly focus on the cervical alignment change and did not analyze the correlation between the muscle change by MRI.

## 5. Conclusion

In conclusion, modified Kurokawa cervical laminoplasty is suitable for patients of CSM with straight cervical alignment. By reconnecting the SPMLC and postoperative muscular exercise, the patients could maintain or improve physiological alignment, prevent postoperation kyphosis deformity, and preserve most of the cervical ROM at 2 years follow-up.

The article "Analysis of Cervical Spine Alignment Change after Modified Kurokawa Cervical Laminoplasty in the Patients with Cervical Myelopathy and Straight Cervical Spine" was published in 2021. Journal: Biomed Res Int.

## Figures and Tables

**Figure 1:** A classification of the cervical alignment proposed by Toyama et al. [10]. According to the relationship of vertebral bodies of C3, C4, C5, and C6 to a virtual straight line drawn from the posteroinferior border of the body of C2 to that of C7, patients were divided into four groups: the lordotic group and the straight, sigmoid, and kyphosis groups. The straight group included patients in whom the posterior cortices of the most anterior and posterior vertebral bodies from C3 to C6 were located within 2 mm either anteriorly or posteriorly from the line.

**Figure 2:** Surgical technique. **(**a) The supraspinous ligament preservation and the connecting points between the posterior muscular ligament complex with the bony elements. (A) The preservation of muscular attachment during the laminoplasty. Just near the medial side of the articular capsular. During the final stage of suturing, we need to connect (B) with (D), (C) with (E) and (F) contralaterally. (b**)** Posterior view of reconnection between the muscular ligament and bonny elements. (c) Adjustment of Mayfield three-point head fixator from the mild straight curve in the beginning of surgery to the lordotic curve in the beginning of suturing. The original distance between C2 and C7 is distance (A); after suturing, the distance changed to (B) (A > B). (C) The continuous suturing of posterior ligament and fascia to form a strong tension bend which could maintain the lordotic curve.

**Figure 3:** Typical case imaging. 42 years female, felt both upper limb numbness and muscle weakness for 2 years. She was diagnosed as cervical spondylosis and treated with double-door laminoplasty. The preoperation JOA score and postoperation JOA score are, respectively, 11 and 15. (a), (b), (c), and (d) were, respectively, lateral view, flexion view, extension view of X-ray, and MRI scan before the surgery. (e), (f), (g), and (h) were, respectively, lateral view, flexion view, extension view, and MRI scan at 2 years follow-up. Angle *α* and *α*1 were cobb angle between C2 and C7. Angle *β* and *β*1 were T1 slope angle. The angle between line AB and CD represent the intervertebral space angle (*α* = −13.3°, *α*1 = 10.6°; *β* = 23.4°, *β*1 = 16.3°; C2 − C7 SVA = 28.6 mm, C2 − C7 SVA1 = 22.1 mm).

**Figure 4:** Comparison of IVD space alignment and ROM according to preoperative T1 Slope.

**Table 1:** Cervical radiological parameter changes.

	Preoperative	2 years follow-up	Change	*P* value
Cervical alignment (°)	1.29 ± 10.04	9.58 ± 8.65	8.29 ± 13.28	0.0098^∗^
C2/3 IVDA (°)	−1.37 ± 4.862	1.71 ± 4.67	3.08 ± 5.05	0.0114^∗^
C3/4 IVDA (°)	−3.87 ± 3.64	−0.65 ± 4.78	3.22 ± 4.23	0.0024^∗^
C4/5 IVDA (°)	−2.06 ± 5.78	1.90 ± 4.87	3.96 ± 7.90	0.0328^∗^
C5/6 IVDA (°)	−0.63 ± 6.39	2.52 ± 4.40	3.15 ± 6.83	0.0477^∗^
C6/7 IVDA (°)	0.86 ± 4.74	1.31 ± 4.23	0.45 ± 6.09	0.7358
ROM	36.8 ± 18.92	25.08 ± 12.10	−11.72 ± 17.33	0.0024^∗^
Flexion C2-7 Cobb angle (°)	−19.90 ± 5.77	−10.00 ± 10.26	10.90 ± 8.78	0.0001^∗^
C2/3 flexion IVDA (°)	−5.54 ± 3.91	−3.46 ± 3.91	2.43 ± 3.71	0.0294^∗^
C3/4 flexion IVDA (°)	−5.82 ± 1.76	−4.04 ± 3.55	2.19 ± 2.84	0.0091^∗^
C4/5 flexion IVDA (°)	−4.35 ± 2.83	−0.66 ± 4.16	3.76 ± 4.35	0.0038^∗^
C5/6 flexion IVDA (°)	−3.98 ± 2.42	−0.38 ± 3.87	3.64 ± 4.24	0.0013^∗^
C6/7 flexion IVDA (°)	−4.21 ± 3.57	−1.62 ± 6.17	2.75 ± 4.74	0.0083^∗^
Extension C2-7 Cobb angle (°)	18.94 ± 17.08	17.87 ± 13.24	−2.86 ± 12.19	0.6561
C2/3 extension IVDA (°)	2.96 ± 3.98	3.02 ± 4.43	−0.24 ± 4.33	0.2050
C3/4 extension IVDA (°)	3.96 ± 4.27	2.61 ± 5.42	−1.61 ± 3.05	0.0394^∗^
C4/5 extension IVDA (°)	3.15 ± 5.99	3.06 ± 3.98	−0.39 ± 4.12	0.9373
C5/6 extension IVDA (°)	2.74 ± 5.26	5.19 ± 4.62	1.93 ± 5.29	0.0579
C6/7 extension IVDA (°)	3.79 ± 5.36	3.31 ± 5.31	−0.81 ± 4.68	0.9851
C2/3 ROM (°)	8.50 ± 3.74	5.84 ± 3.79	−2.67 ± 6.03	0.0094^∗^
C3/4 ROM (°)	9.92 ± 3.19	5.99 ± 4.01	−3.93 ± 3.02	<0.0001^∗^
C4/5 ROM (°)	7.50 ± 6.71	3.35 ± 3.25	−4.15 ± 6.11	0.0236^∗^
C5/6 ROM (°)	6.64 ± 5.34	5.02 ± 3.11	−1.62 ± 4.24	0.2035
C6/7 ROM (°)	8.00 ± 4.63	4.44 ± 3.72	−3.56 ± 5.21	0.0183^∗^
T1 slope angle (°)	22.25 ± 6.28	20.71 ± 3.78	−1.54 ± 4.14	0.1036
T1 slope flexion angle (°)	30.87 ± 10.2	30.52 ± 11.66	−3.40 ± 17.03	0.9749
T1slope extension angle (°)	21.20 ± 5.92	17.61 ± 7.51	−5.35 ± 11.04	0.1447
Neutral C1-2 angle (°)	31.33 ± 6.26	34.48 ± 6.22	3.15 ± 4.59	0.0052^∗^
Flexion C1-2 angle (°)	23.54 ± 10.92	21.33 ± 7.88	−4.34 ± 11.11	0.3521
Extension C1-2 angle (°)	31.03 ± 5.99	33.21 ± 5.82	−1.14 ± 11.65	0.0361^∗^
C2-C7 SVA (mm)	28.5 ± 3.2	22.6 ± 6.7	−6.7 ± 1.3	0.0113^∗^

The data was presented as mean ± SD, “^∗^” means *P* < 0.05, and there was a significant statistical difference between different time points.

The article "Analysis of Cervical Spine Alignment Change after Modified Kurokawa Cervical Laminoplasty in the Patients with Cervical Myelopathy and Straight Cervical Spine" was published in 2021. Journal: Biomed Res Int.

**Table 2:** Correlation analysis.

Factor A	Factor B	*r*	*P* value
C1/2 angle change	Cervical alignment change	-0.4499	0.0465^∗^
Preoperative C1/2 angle	Preoperative cervical alignment	-0.7859	<0.0001^∗^
Postoperative C1/2 angle	Postoperative cervical alignment	-0.4771	0.0334^∗^
C2/4 angle change	Cervical alignment change	0.8086	0.0046^∗^
C2/4 ROM change	ROM change	0.2484	0.291
Preoperative T1 slope	Preoperative cervical alignment	0.3972	0.0297^∗^
Postoperative T1 slope	Postoperative cervical alignment	0.4063	0.0259^∗^
Preoperative T1 slope	Preoperative NFRROM	0.2251	0.2317
Postoperative T1 slope	Postoperative NFRROM	0.4507	0.0124^∗^
C2-C7 SVA change	Cervical alignment change	-0.3442	0.0015^∗^
Preoperative cervical alignment	Preoperative NFRROM	0.1085	0.5684
Postoperative cervical alignment	Postoperative NFRROM	0.5171	0.0034^∗^

“^∗^” means *P* < 0.05, and there was significant correlation between the factors.

## Data Availability

The data are available on request.
